# Molecular signaling pathways in osteoarthritis and biomaterials for cartilage regeneration: a review

**DOI:** 10.1080/21655979.2025.2501880

**Published:** 2025-05-07

**Authors:** Samson Prince Hiruthyaswamy, Arohi Bose, Ayushi Upadhyay, Tiasa Raha, Shangomitra Bhattacharjee, Isheeta Singha, Swati Ray, Nazarene Marylene Nicky Macarius, Pragasam Viswanathan, Kanagavel Deepankumar

**Affiliations:** Department of Biotechnology, School of Biosciences and Technology, Vellore Institute of Technology, Vellore, India

**Keywords:** Osteoarthritis, biomaterials, CRISPR/Cas9, molecular pathways, cartilage regeneration, inflammation

## Abstract

Osteoarthritis is a prevalent degenerative joint disease characterized by cartilage degradation, synovial inflammation, and subchondral bone alterations, leading to chronic pain and joint dysfunction. Conventional treatments provide symptomatic relief but fail to halt disease progression. Recent advancements in biomaterials, molecular signaling modulation, and gene-editing technologies offer promising therapeutic strategies. This review explores key molecular pathways implicated in osteoarthritis, including fibroblast growth factor, phosphoinositide 3-kinase/Akt, and bone morphogenetic protein signaling, highlighting their roles in chondrocyte survival, extracellular matrix remodeling, and inflammation. Biomaterial-based interventions such as hydrogels, nanoparticles, and chitosan-based scaffolds have demonstrated potential in enhancing cartilage regeneration and targeted drug delivery. Furthermore, CRISPR/Cas9 gene editing holds promise in modifying osteoarthritis-related genes to restore cartilage integrity. The integration of regenerative biomaterials with precision medicine and molecular therapies represents a novel approach for mitigating osteoarthritis progression. Future research should focus on optimizing biomaterial properties, refining gene-editing efficiency, and developing personalized therapeutic strategies. The convergence of bioengineering and molecular science offers new hope for improving joint function and patient quality of life in osteoarthritis management.

## 1. Introduction

Osteoarthritis (OA) refers to a prevalent, age-related, diverse set of illnesses described pathologically by discrete regions of articular cartilage loss in synovial joints, as well as various degrees of osteophyte development, subchondral bone alteration, and synovitis. OA is a commonly occurring condition associated with aging, affecting approximately 10–15% of the global population over the age of 60 and nearly 500 million people worldwide. In the United States alone, 32.5 million adults are affected, making OA one of the leading causes of disability. It encompasses a range of diseases characterized by the pathological loss of articular cartilage in synovial joints, along with the development of osteophytes, changes in subchondral bone, and inflammation of the synovial membrane. Joint damage is caused by a combination of systemic characteristics that increase an individual’s susceptibility to the disease and local mechanical factors that determine the extent and progression of the injury [1]. Osteoarthritic joint degeneration is linked to clinical problems; however, there is a weak relationship between the degree of joint disease and the severity of clinical symptoms [2]. The progression of OA is frequently gradual, but due to the limited regenerative capacity of cartilage, it ultimately results in the deterioration of joint function. Several risk factors have been associated with OA, including aging, mechanical stress, obesity, genetic predisposition, and traumatic joint injury. Despite extensive research, the exact underlying cause of OA remains unknown, and an effective cure has yet to be discovered [3].

The pathological changes associated with OA include articular cartilage fibrillation, thickening of the subchondral bone, production of osteophytes, inflammation of the synovium, degeneration of the ligaments, and hypertrophy of the joint capsule [4]. Severe cases show subchondral sclerosis and cysts on radiographs, along with microfractures and microcracks on microscopic examination. Maintaining chondrocyte homeostasis is key; disruptions lead to cartilage degradation. Understanding these mechanisms is vital for targeted therapeutic development and cartilage [5]. Presently, there’s no cure for OA, necessitating ongoing management. Recent advances in osteogenesis and bone regeneration have highlighted the role of functional biomaterials in promoting tissue repair. Biomaterials such as hydrogels, nanomaterials, and bioengineered scaffolds have demonstrated significant potential in OA treatment by enhancing cell proliferation and extracellular matrix synthesis [6]. Additionally, electrospun fiber-based immune engineering has emerged as a promising strategy in regenerative medicine, where nanofiber scaffolds facilitate immune regulation and support cartilage regeneration [7]. Beyond OA treatment, biomaterials have been extensively explored in reconstructive surgery and regenerative medicine, showcasing their versatility. For example, Asian facial recontouring surgery and alveolar cleft reconstruction with vomerine bone grafting have demonstrated novel applications of biomaterials for tissue engineering [8–10]. Moreover, blood-derived biomaterials, such as platelet-rich plasma (PRP), have shown promise in wound healing, cosmetic procedures, and fat grafting, though further standardized trials are required to validate their efficacy. The growing demand for facial rejuvenation treatments, including invasive and noninvasive procedures, has also fueled advancements in biomaterials, with noticeable variations in treatment preferences. The CRISPR/Cas system offers a promising avenue, allowing precise genome manipulation for tackling this condition. In healthy cartilage, chondrocytes maintain a delicate balance between anabolic and catabolic processes, disrupted by aging and joint degeneration. Understanding these mechanisms is crucial for targeted therapeutic development, aiming at biological approaches for cartilage regeneration in OA and related joint disorders [11]. These advancements reinforce the significance of biomaterials and regenerative medicine in orthopedic, reconstructive, and aesthetic applications, emphasizing the need for continued interdisciplinary collaboration among experts in biology, clinical medicine, and biomaterial sciences.

The primary focus of this review is on the fundamental mechanisms underlying cartilage physiopathology. The main signals that can initiate cellular and molecular processes in cartilage degradation and regeneration will be discussed in detail. Understanding these mechanisms is essential for developing biological strategies to enhance cartilage regeneration and identifying important pathogenic factors as specific therapeutic targets.

## 2. Osteoarthritis and its pathogenesis

Normal bone maintains its structure and density, with a smooth surface and healthy cartilage covering the ends of bones at joints. Joint cartilage, or articular cartilage, is a specialized connective tissue that lines the ends of bones in synovial joints, providing a smooth, lubricated surface for movement while distributing mechanical loads to minimize stress on bones during motion. The extracellular matrix (ECM) of cartilage is highly resilient, primarily composed of water, collagen fibers, and proteoglycans. This unique composition enables cartilage to withstand compressive forces and serve as an effective cushion within the joint. The cellular component of cartilage consists predominantly of chondrocytes, the specialized cells responsible for synthesizing and maintaining the ECM. These cells are embedded within small cavities called lacunae, where they produce essential structural components such as collagen and proteoglycans to preserve cartilage integrity and function [12–14]. Additionally, chondrocytes regulate cartilage metabolism by responding to mechanical signals and maintaining tissue homeostasis, ensuring the joint remains functional and resilient under varying load conditions. In contrast, OA affects bone by causing the breakdown of cartilage, resulting in rough and uneven surfaces. The result of this disintegration may be the development of osteophytes, or bone spurs, around the affected joint shown in Figure 1. Additionally, OA can cause changes in bone density, with areas of increased density (sclerosis) near the joint surface and cyst formation within the bone. Overall, osteoarthritic bone exhibits structural changes and alterations in density compared to normal bone. Early OA stages involve proteoglycan depletion and collagen disarray. As degradation progresses, cartilage ulceration releases proteoglycans into synovial fluid, reducing cartilage water content. Later stages are marked by significant loss in collagen, proteoglycan, and water content. Furthermore, the collagen network experiences major disruption [15]. The knee joint’s stability relies on various structures. Articular cartilage, rich in type II collagen and proteoglycans, facilitates smooth joint movement and load distribution. The underlying subchondral bone, composed of mineralized type I collagen, provides mechanical support and absorbs shock. The menisci, with their water-rich collagen-proteoglycan composition, act as crucial shock absorbers, dampening mechanical forces and reducing joint stress. The synovial membrane plays a key role in joint lubrication by secreting synovial fluid, which contains essential components such as hyaluronic acid and lubricin. However, in OA, these protective mechanisms deteriorate, leading to increased mechanical stress and cartilage breakdown. The weakening of the menisci, coupled with chronic synovial inflammation, contributes to meniscal tears and progressive cartilage erosion. The loss of cartilage integrity increases friction between joint surfaces, further accelerating damage. Notably, in the early stages of OA, proinflammatory cytokines such as interleukin − 1 β (IL-1β) and tumor necrosis factor - α (TNF-α) drive synovial inflammation and matrix degradation, exacerbating cartilage destruction and joint dysfunction [16].

**Figure 1.** Cytokine-mediated inflammation and osteophyte formation in OA.

### 2.1. Articular cartilage and the impact of mechanical loads

Articular cartilage is a thin, stretchable, load-bearing tissue that lines the bone extremities of diarthrodial joints. Its primary functions include stabilizing and guiding joint motion while distributing forces that occur during joint loading [17]. Additionally, it plays a crucial role in joint lubrication. When external forces are applied, the cartilage deforms, expanding joint contact regions and reducing contract stresses. This response is highly specific due to its unique composition and structural properties [18]. Mechanical loading is essential for maintaining cartilage health and functionality. Inadequate loading can lead to cartilage atrophy, as regular mechanical stimulation is necessary to preserve proteoglycan content, a key component of the extracellular matrix. Reduced loading results in decreased proteoglycan levels, weakening the cartilage and increasing susceptibility to degeneration. Furthermore, chondrocytes, responsible for cartilage maintenance, rely on mechanical signals for proper function. Without adequate stimulation, chondrocyte activity declines, impairing cartilage repair and regeneration. Conversely, excess mechanical stress caused by overweight and obesity accelerates cartilage wear, particularly in weight-bearing joints like the knees and hips. Excess body weight significantly increases joint loading, with each pound of weight exerting approximately four pounds of pressure on the knees. This heightened stress contributes to faster cartilage breakdown and OA progression. Additionally, obesity is linked to systemic inflammation, as adipose tissue releases pro-inflammatory cytokines that exacerbate joint inflammation and cartilage degradation. Both inadequate mechanical loading and excessive weight negatively impact cartilage health, highlighting the importance of maintaining a healthy weight and engaging in regular physical activity to reduce the risk of OA [19,20].

### 2.2. Chondrocyte dysfunction

Mitochondria play a crucial role in regulating cellular function and viability, significantly influencing the onset and progression of age-related diseases, including OA. Age-related modifications in mitochondrial function have been linked to accumulated mutations in mitochondrial DNA (mtDNA) and prolonged exposure to oxidative stress, both of which contribute to cellular dysfunction. Articular cartilage, composed of chondrocytes embedded in an extracellular matrix, relies on mitochondrial activity for energy production and redox balance. However, in OA, mitochondrial dysfunction leads to excessive production of reactive oxygen species (ROS), causing oxidative damage to cellular components. This oxidative stress disrupts chondrocyte homeostasis, triggering inflammatory responses and enhancing the activity of matrix-degrading enzymes such as matrix metalloproteinases (MMPs) and aggrecanases. Therefore, chondrocytes undergo apoptosis, a programmed cell death process that results in a progressive decline in cell population. The loss of viable chondrocytes impairs extracellular matrix maintenance and accelerates cartilage degradation. This decline in cartilage integrity further exacerbates joint dysfunction, contributing to OA progression. Understanding the role of mitochondrial dysfunction in chondrocyte apoptosis provides critical insights into potential therapeutic strategies aimed at preserving cartilage health and delaying OA-related joint deterioration [21–23].

### 2.3. The function of inflammation in osteoarthritis

OA is a joint condition characterized by inflammation, which is a key defense mechanism against infection. Factors such as genetic susceptibility, joint mechanical load, and inflammation can contribute to its progression [24,25]. In individuals with end-stage OA, synovial fluids contain higher levels of proinflammatory cytokines and chemokines. Chondrocytes, typically dormant cells, release proinflammatory cytokines, causing collagenases and aggrecans to break down cartilage as illustrated in Figure 1 [26,27]. In addition to releasing cytokines like interleukin-6 (IL-6) and IL-1β, activated immune cells like neutrophils and macrophages can also exacerbate inflammation. OA also increases the infiltration of leukocytes in the synovium, particularly in the subintimal layer. Treatment targets cytokines TNF-α, interleukin-1 (IL-1), and IL-6, which are generated by chondrocytes, synoviocytes, macrophages, and osteoblasts [28–30].

### 2.4. Osteophyte formation

Osteophytes are a characteristic of OA that are osseocartilaginous outgrowths near the margins of joints. They are derived from adult knee Gdf5-expressing embryonic joint interzone cells, which support cartilage regeneration and synovial hyperplasia. In the early stages of development, human osteophytes in OA hip and knee joints express osteocalcin and have endochondral bone coated in a cartilage cap. In OA, progenitor cell subsets that reside in the joint respond to cues and cooperate to become osteophytes [31,32]. A study by Ikufumi Takahashi et.al examined the histological effects of knee loading reduction on osteophyte development, synovitis, and cartilage degradation in early-stage OA. The study found that decreased knee joint stress significantly slowed the course of OA [33].

### 2.5. OA anti-inflammatory drugs

Osteoarthritis management involves non – steroidal anti-inflammatory drugs (NSAIDs) like ibuprofen for pain relief, though long-term use poses risks. Corticosteroid and hyaluronic acid injections offer temporary relief but may impact cartilage health. Biologic agents such as TNF-α and IL-1 inhibitors target inflammation, while disease-modifying drugs like sprifermin and licofelone aim to slow progression. Opioids provide severe pain relief but carry dependency risks. Nutraceuticals like glucosamine and omega-3s have mixed evidence. Emerging therapies, including monoclonal antibodies, PRP, and stem cells, hold promise. A multimodal approach combining pharmacological treatments, physical therapy, and regenerative medicine is essential for effective OA management [34]. In OA patients, IL-1 expression has been widely observed in the cartilage, synovium, and synovial fluid (SF). Genetic recombination produces drugs that target the IL family, such as Anakinra and the monoclonal antibody AMG 108, which targets the human IL-1 receptor type 1. TNF-α, which is generated by chondrocytes and synoviocytes in OA, is essential for controlling pain and structural damage [35,36]. Not only does TNF-α stimulate the production of nitric oxide (NO) and MMP, but it also plays a major role in increasing the production of proinflammatory cytokines including IL-6 and IL-8 [36]. One such drug is the fusion protein known as etanercept, which is a recombinant human necrosis factor type II antibody. According to studies, etanercept injections, a TNF-α inhibitor, have been found to effectively reduce pain in OA patients compared to high molecular weight hyaluronic acid injections. This suggests that TNF-α plays a crucial role in OA-related pain and inflammation. In addition to etanercept, other TNF-α inhibitors, such as Infliximab and Adalimumab, are being evaluated for their potential benefits in OA treatment. While clinical studies on Infliximab’s efficacy in OA remain limited, its role in reducing systemic inflammation warrants further investigation. Beyond TNF-α inhibition, specialized pro-resolving mediators like resolvin D1 (RvD1), derived from omega-3 fatty acids, have shown promising anti-inflammatory and anti-apoptotic effects in OA. RvD1 helps regulate immune responses, reduce synovial inflammation, and protect chondrocytes from apoptosis, offering an additional therapeutic avenue for managing OA symptoms [37–39].

## 3. Osteoarthritis and its pathways

OA progresses through several stages, including pre-osteoarthritis, early, mild, moderate, and severe phases. At the molecular level, traumatic injury triggers mechanical imbalance and overload, setting off multiple inflammatory signaling pathways, including poly adenosine diphosphate (ADP)-ribose (PAR)-synoviocytes, cyclooxygenase-2 (COX-2), inducible nitric oxide synthase (iNOS), and nuclear factor kappa B (NF-kB), all of which contribute to cartilage degeneration. Understanding chondrogenesis, the process by which cartilage develops and matures, provides insight into potential therapeutic interventions. Chondrogenesis progresses through four main stages: condensation, proliferation and differentiation, maturation, and terminal differentiation as shown in Figure 2. In the condensation phase, mesenchymal stem cells (MSCs) aggregate and are primed for differentiation under the influence of TGF-β, BMP-2, BMP-4, BMP-7, FGF-2, Sonic Hedgehog (Shh), and Wnt-3a, with Sox9 acting as a key transcription factor initiating chondrogenesis. During proliferation and differentiation, chondroprogenitors expand and differentiate into chondroblasts, driven by IGF-1, FGF-2, BMP-2, BMP-4, and BMP-7, while Sox9, Sox5, and Sox6 coordinate cartilage-specific gene expression. As the process advances to differentiation and maturation, chondrocytes develop and produce extracellular matrix components essential for cartilage formation, regulated by BMP-2, VEGF, FGF-2, Wnt-4, Wnt-8, and β-catenin, with Sox9, Sox5, and Sox6 maintaining cartilage integrity. Finally, in terminal differentiation, chondrocytes undergo hypertrophy, contributing to cartilage calcification and bone formation, a transition controlled by Runx2, Osterix, and TCF/LEF-1, which promote matrix remodeling and mineralization. This intricate interplay of molecular signals governs cartilage formation and highlights potential therapeutic targets for osteoarthritis intervention.

**Figure 2.** Stages of chondrogenesis and key regulatory factors.

### 3.1. FGF pathway

Cartilage degeneration in OA and degenerative disc disease can be targeted for therapy by investigating molecular mechanisms involving FGF-2, FGF-18, and FGF-8, as shown in Figure 3, which highlights their crucial roles in cartilage health. Figure 3 illustrates a signaling pathway involved in cartilage repair, emphasizing the role of FGFR3 (Fibroblast Growth Factor Receptor 3) in regulating cartilage metabolism and inflammation. The pathway begins with Indian Hedgehog (IHH), a key regulator of cartilage development, whose activity is inhibited by GDC0449, an IHH inhibitor. This inhibition affects the downstream activation of FGFR3, which plays a crucial role in cartilage homeostasis. FGFR3 is activated by high-affinity ligands such as FGF9 or FGF18 and is further influenced by FGF2, FGF21, and FGF23, all of which contribute to cartilage maintenance. Once activated, FGFR3 regulates several critical processes, including extracellular matrix (ECM) production, which is essential for maintaining cartilage integrity. Additionally, it modulates pro-inflammatory mediators, helping control inflammation in the joint environment, while also regulating matrix metalloproteinases (MMPs), enzymes responsible for cartilage degradation. Furthermore, FGFR3 plays a role in hypertrophic differentiation, a process affecting the growth and repair of cartilage cells. Ultimately, these molecular interactions contribute to cartilage repair, highlighting the potential of targeting FGFR3-related pathways for therapeutic interventions in conditions such as OA and cartilage injuries.

**Figure 3.** Fibroblast growth factors in cartilage homeostasis and OA.

These fibroblast growth factors (FGFs) regulate OA progression and cartilage homeostasis through their respective receptors, fibroblast growth factor receptor 1 (FGFR1) and fibroblast growth factor 3 (FGFR3). FGF-2 primarily interacts with FGFR1, leading to the upregulation of MMPs and aggrecanases, which promote cartilage degradation. Excessive FGF-2 activity inhibits proteoglycan synthesis and contributes to chondrocyte clustering, a hallmark of OA pathology. In contrast, FGF-18 exerts an anabolic effect via FGFR3, enhancing ECM production, type II collagen synthesis, and chondrocyte proliferation, which facilitate cartilage repair. Meanwhile, FGF-8, also linked to FGFR1, plays a catabolic role in OA progression by stimulating MMP-13, an enzyme responsible for cartilage breakdown [40]. FGF-2’s impact on cartilage varies across species and age, with recent findings suggesting it may negatively influence human cartilage and intervertebral disc tissue by activating FGFR1 [41]. Increased production of ECM degradation enzymes, inhibited ECM buildup and proteoglycan synthesis, and cell clustering are associated with arthritis. In articular cartilage ECM, a proteoglycan called perlecan binds FGF-2, which is produced in cartilage. Upon cartilage damage, released FGF-2 activates the ERK pathway. However, varied species studies yield inconsistent conclusions regarding FGF-2’s role in ECM synthesis and cartilage homeostasis [42]. FGF-2 has anti-catabolic effects on cartilage in vitro, as it increases TIMP1 expression in mouse cartilage and decreases a disintegrin and metalloproteinase with thrombospondin motifs 4 (ADAMTS4) and (ADAMTS5) activity in human cartilage induced by IL-1. Additionally, FGF-2 promotes mitogenic effects, aiding articular cartilage regeneration in vivo in rabbit knee injuries [43]. The significance of FGF-2 in maintaining mouse articular cartilage is evident, as complete isoform ablation accelerates OA development, which is reversible with recombinant FGF-2. Interestingly, certain studies show that low molecular weight (LMW) FGF-2 isoform ablation offers protection against OA [44].

FGF-1 also plays a role in OA pathogenesis. Serum FGF-1 levels correlate positively with early-stage knee OA radiographic features, while its increased production in the synovial membrane is associated with late-stage OA development [41]. In a rat OA model, FGF-1 is induced in articular cartilage, and FGF-1 therapy in human chondrocytes increases MMP13 expression while suppressing aggrecan and type II collagen expression. Additionally, FGF-1 inhibits cellular communication network factor 2, suggesting catabolic effects on chondrocytes [45,46]. FGF-18, acting via FGFR3c, exhibits protective roles in OA. It is significantly expressed in the superficial zone of mouse cartilage, which is home to stem/progenitor cells. FGF-18 is an anabolic factor that preserves glycosaminoglycan in cartilage, essential for synovial joint formation, by upregulating TIMP1 expression [47]. It enhances type II collagen and proteoglycan accumulation in porcine and human chondrocytes, promotes chondrogenesis, and aids cartilage repair in OA rat models. Furthermore, FGF-18 acts as a protective factor, safeguarding articular cartilage from degeneration [40]. In contrast, FGF-8 has been associated with cartilage degeneration in some animal studies, though its exact effects on adult human cartilage and intervertebral disc (IVD) tissue remain unclear. Current evidence suggests targeting FGF-8 with antagonists, such as anti-FGF-8 antibodies, as a potential therapeutic strategy for cartilage degeneration. Additionally, FGF-2/FGFR1 inhibition has been proposed as another promising therapeutic approach [43]. Other FGFs may also contribute to cartilage homeostasis. Reduced FGF-9 expression in human OA cartilage suggests a potential protective role similar to FGF-18. Exogenous FGF-9 treatment in mouse post-traumatic OA models reduces cartilage degradation and enhances osteophyte development, though further human studies are needed to confirm its role in clinical OA management [48]. Meanwhile, FGF-7 and FGF-10, possibly acting via FGFR1b and FGFR2b, have been implicated in OA pathogenesis. Exogenous FGF-10 application leads to fusion of cartilaginous phalanges in chick limb buds, suggesting its involvement in joint development and repair [42].

### 3.2. Akt Pathway

The Akt pathway, vital for cell survival, proliferation, and differentiation, is crucial in OA pathophysiology. Phosphatidylinositol 3-kinase (PI3K), activated at the cell membrane, converts PIP2 to PIP3, initiating Akt signaling, pivotal in OA’s inflammatory and cartilage degradation processes. PIP3 is phosphorylated by mammalian target of rapamycin complex 2 (mTORC2) and the phosphoinositide-dependent kinase 1 (PDK1). This process recruits and activates Akt, which is sometimes referred to as protein kinase B (PKB) [49]. In OA, pro-inflammatory cytokines and enzymes that break down cartilage are induced by the nuclear factor-kappa B (NF-κB), which is regulated by Akt pathway. It promotes cell survival, inhibiting apoptosis that contributes to cartilage breakdown. Akt also modulates MMP activity, aiding cartilage matrix formation, and reduces inflammation by inhibiting inflammatory molecule production [50]. The diverse roles of the Akt pathway in OA highlight its significance as a research and treatment target. Further investigation is vital to understand its therapeutic potential fully, considering its context-dependent functions across different cellular environments and disease stages [52].

The activation of receptors is a crucial component of the Akt pathway, which governs several downstream signaling pathways involved in OA progression, as illustrated in Figure 4, where pro-inflammatory molecules and catabolic enzymes (e.g. MMPs, cytokines) are highlighted in red, signifying their destructive effects on cartilage. Signaling molecules (e.g. PI3K, Akt, PIP3) are shown in blue, emphasizing their role in cellular communication and metabolic regulation. Meanwhile, protective or anti-apoptotic components (e.g. survival-promoting factors) appear in green, highlighting their function in chondrocyte survival and ECM maintenance. The phosphoinositide 3-kinase (PI3K)/Akt/mammalian target of rapamycin (mTOR) pathway plays a key role in chondrocyte survival, cartilage metabolism, and inflammation in OA [51]. Upon activation, PI3K converts phosphatidylinositol-4,5-bisphosphate (PIP2) into phosphatidylinositol-3,4,5-triphosphate (PIP3), triggering Akt phosphorylation. Activated Akt regulates matrix metalloproteinases (MMPs), apoptosis inhibition, and inflammatory cytokine production, all of which influence cartilage degradation and joint inflammation.

**Figure 4.** PI3K/Akt/mTOR pathway in OA.

Growth factor receptors, including cytokine receptors and insulin-like growth factor-1 (IGF-1), are linked to Akt activation. PIP3 recruits PI3K, a crucial regulator of protein synthesis and cell proliferation, to the cell membrane as a second messenger. There, it is phosphorylated by mTORC2 and phosphoinositide-dependent kinase 1 (PDK1) [52]. Akt signaling inhibits chondrocyte apoptosis, crucial in OA pathogenesis, and promotes cartilage matrix synthesis via anabolic pathways, aiding in collagen and proteoglycan production. Akt also helps maintain cartilage homeostasis in response to mechanical stress, while dysregulated MMP activity contributes to OA cartilage degeneration [53]. In addition to having anti-inflammatory properties, Akt activation can help manage OA by lowering the production of pro-inflammatory mediators. The Akt pathway’s significance in OA arises mostly from its function in controlling the activity of chondrocytes, or cartilage cells and maintaining the homeostasis of cartilage [54]. The Akt pathway, vital for cartilage integrity, shields chondrocytes from apoptosis in OA. It inhibits pro-inflammatory substances and promotes anabolism. However, dysregulated Akt activation can degrade cartilage via excessive catabolic enzyme synthesis exacerbated by mechanical stress. Factors such as obesity and joint injury can contribute to this. Aging also affects the Akt pathway’s activity, affecting osteoarthritis development and progression.

### 3.3. BMP pathway

The bone morphogenetic protein (BMP) pathway plays a crucial role in regulating bone and cartilage homeostasis, with its dysregulation being strongly associated with OA. BMPs, a group of growth factors within the transforming growth factor-beta (TGF-β) superfamily, are essential for bone development, repair, and remodeling. This pathway contributes to both joint tissue maintenance and pathological changes, as illustrated in Figure 5. In healthy cartilage, BMP-2 and BMP-7 activate the Smad 2/3 complex, which binds to Smad4 and translocates to the nucleus, upregulating the expression of type II collagen (Col2a1) and aggrecan (ACAN) – two key components that maintain ECM integrity and ensure cartilage health. However, excessive BMP signaling can contribute to OA progression by upregulating Indian hedgehog (Ihh) and runt-related transcription factor 2 (Runx2), which drive chondrocyte hypertrophy, osteophyte formation, and subchondral bone sclerosis – hallmarks of OA pathology. Additionally, BMP signaling interacts with Wnt/β-catenin and PI3K/Akt pathways, further influencing chondrocyte survival, inflammation, and cartilage degradation.

**Figure 5.** Bone morphogenetic protein signaling in cartilage maintenance and OA progression.

A study led by Liu and colleagues aimed to investigate the function of bone morphogenetic protein 9 (BMP9) in the chondrogenic development of mesenchymal stem cells generated from adipose tissue (ADMSCs). They evaluated Type II collagen and aggrecan expressions using RT-qPCR, western blotting, and BMP9 mRNA expression. For the experiment, mice with osteoarthritis were employed. An intra-articular injection of ADMSCs overexpressing BMP9 was administered to the OA-affected knee joint [55]. Using western blot analysis and RT-qPCR, the researchers then investigated the intra-articular expression of Type II collagen and aggrecan. They also measured the expression levels of Notch1 and Jagged1, two proteins linked to the Notch signaling pathway [55,56]). The overexpression of BMP9 enhances the expression of Type II collagen and aggrecan and is essential for the differentiation of ADMSCs into chondrogenic tissue. Moreover, BMPs activate SMAD proteins, which are intracellular mediators crucial for gene regulation in chondrogenesis and osteogenesis [57]. The healing of cartilage in knee joints damaged by OA was reduced when Notch signaling was inhibited in ADMSCs (Hosaka et al., 2013). This shows that chondrogenic development in ADMSCs can be improved by upregulating BMP9 protein expression. BMP signaling also interacts with Indian Hedgehog (Ihh) pathways, influencing the differentiation of mesenchymal cells into chondrocytes [58]. In knee joints damaged by OA, intraarticular injection of ADMSCs via the Notch1/Jagged1 signaling pathway facilitates cartilage healing. BMP signaling upregulates Runx2, essential for osteoblast differentiation, promoting the differentiation of mesenchymal stem cells into osteoblasts [59]. An inhibitor of the Notch signaling system, LY411575, dramatically reduced the development of cartilage in ADMSCs [55]. Furthermore, BMP signaling enhances the expression of collagen, particularly Type II collagen in chondrocytes and Type I collagen in osteoblasts, important for maintaining the extracellular matrix in cartilage and bone [60]. Liao et al. sought to determine if osteogenesis and angiogenesis coupling in MSCs was improved by concurrent stimulation of the BMP9 and Notch pathways [61]. In their investigation, MSCs were derived from immortalized mouse adipose-derived progenitor cells (MADS). Adenoviral vectors introduced transgenes dnNotch1, NICD, and BMP9. Immunohistochemistry and qPCR quantified gene expression. BMP9 increased Notch receptor and ligand expression in iMADs [62]. In vitro and in vivo BMP9-induced osteogenic differentiation was markedly amplified by the constitutively active expression of Notch1, NSD1. Addition of dominant-negative Notch1, dnNotch1, effectively inhibited this increase [63]. MSCs transduced with BMP9 and NICD1 generated fully mature bone tissue with notable blood vascular development when implanted with a biocompatible scaffold [64]. Significantly elevated by NICD1, while dnNotch1 was inhibited, important angiogenic regulators produced by BMP9 in iMADS and VEGFA in the ectopic bone [61]. BMPs like BMP-2 and BMP-7 are potential disease-modifying agents for OA due to their roles in cartilage homeostasis and repair. They enhance collagen and proteoglycan production, stimulate anabolic responses in chondrocytes, facilitate chondroprogenitor recruitment, and demonstrate chondroprotective effects in OA animal models [65,66].

## 4. Biomaterial-based cartilage repair

### 4.1. Biomaterials and their molecular pathways in osteoarthritis treatment

Certain polymers used in fabricating adhesive hydrogels exhibit inherent biological functions, contributing significantly to OA therapy. Key functional components include hyaluronic acid (HA), gelatin, alginate, and chondroitin sulfate (CS), as outlined in Table 1, which summarizes their respective molecular pathways. The concentration of hyaluronic acid in the synovial fluid of osteoarthritic joints is typically lower compared to that in healthy joints. As a result, the FDA has approved intra-articular HA injections as a treatment for OA due to their ability to enhance joint lubrication and reduce inflammation [70]. HA plays a key role in suppressing the production of inflammatory mediators such as IL-1β, IL-6, and TNF-α, while also inhibiting matrix metalloproteinases (MMPs) and prostaglandin E2 (PGE2) synthesis via CD44 receptor interactions. Additionally, HA downregulates p65 NF-κB and IκBα phosphorylation, which are activated by lipopolysaccharides (LPS) through the intercellular adhesion molecule-1 (ICAM-1) receptor [67]. Studies using pig models have demonstrated that HA not only preserves the chondrogenic phenotype but also modifies the trabecular structure of subchondral bone, reducing cartilage stress caused by mechanical impact [85]. Furthermore, HA facilitates cell migration and angiogenesis, contributing to tissue regeneration in a dose-dependent manner [70,86]. Incorporating HA into adhesive hydrogels enhances its biological benefits, making it a promising component for OA treatment [87]. Gelatin, a structural protein derived from collagen hydrolysis, is widely used in regenerative medicine due to its low immunogenicity and bioactive properties. It contains the arginine-glycine-aspartic acid (RGD) sequence, which promotes cell adhesion, proliferation, and differentiation [88]. Recent findings indicate that gelatin-based substrates promote chondrogenesis in bone marrow mesenchymal stem cells (MSCs), as evidenced by increased staining of chondrogenic markers [89]. Similarly, alginate, a naturally occurring polymer, plays a role in extracellular matrix (ECM) mineralization in vitro [90]. Research on animal models has shown that alginate-gelatin scaffolds exhibit excellent mechanical and relaxation properties, providing a suitable microenvironment for ECM remodeling and stimulating cartilage differentiation [74,91–93].

**Table 1.** Biomaterials and their molecular pathways in hydrogel-based OA treatment.

Biomaterials	Biological function	Molecular pathways	Reference
HA	Anti-inflammation; Pain relief.	Interacts with TLR-2 and TLR-4, leading to a decrease in TNF, IL-1β, IL-17, MMP-13, and iNOS	[67–69]
	Chondrogenesis; Inhibition of degradation; Adaptation to mechanical stress	Binds to ICAM-1, suppressing NF-κB and IL-1β; Interacts with CD44, reducing PGE2 while increasing HSP70	[68]
	Promotion of angiogenesis	Through CD44 binding, it downregulates IL-1β, which in turn reduces MMP-1, 2, 3, 9, and 13	[70,71]
	Improvement of cell proliferation	N/A	[71,72]
Gelatin	Cell proliferation	N/A	[73]
Alginate	Aids in adapting to mechanical stress	N/A	[74]
	Stimulates cell proliferation	N/A	[74,75]
Chondroitin Sulphate	Reduces inflammation, relieves pain, and enhances cell growth	Suppresses p38 MAPK and ERK1/2 signaling pathways	[76–79]
Collagen	Supports cartilage formation and reduces inflammation	Encourages T regulatory cell migration and anti-inflammatory cytokine production	[80]
Chitosan	Exhibits tissue adhesion, antioxidant activity, and antibacterial properties	N/A	[81]
Mussel adhesive proteins (MAP)	Tissue adhesion; Cell adhesion	Facilitates DOPA-mediated interfacial bonding	[82,83]
Fibrin glue	Tissue adhesion; Cell delivery	Relies on fibrinogen-thrombin interactions	[84]

Another crucial ECM component, chondroitin sulfate (CS), is essential for maintaining the microstructure and mechanical integrity of the meniscus. A decline in glycosaminoglycan (GAG) content and collagen fiber organization compromises impact absorption and cartilage stability, accelerating OA progression [94]. Furthermore, metabolic alterations in osteoarthritic chondrocytes result in a shift from oxidative phosphorylation to anaerobic glycolysis, triggered by nutrient stress. This transition leads to the inhibition of 5’-AMP-activated protein kinase (AMPK) signaling, intensifying pro-catabolic responses to IL-1β and TNF-α, ultimately promoting cartilage degradation [22]. Additionally, chronic hyperglycemia is linked to the excessive accumulation of advanced glycation end products (AGEs) in joint tissues, which contributes to joint contracture development [95]. Notably, highly purified CS has demonstrated the ability to suppress p38 mitogen-activated protein kinase (MAPK) and extracellular signal-regulated kinase 1/2 (ERK1/2) phosphorylation following stimulation by IL-1β, NF-κB, TNF-α, cyclooxygenase-2 (COX-2), and inducible nitric oxide synthase (iNOS) [76,95]. This inhibition helps alleviate inflammation caused by metabolic and mechanical imbalances, ultimately decelerating OA progression. Research on pig models further confirms that CS incorporation into 3D fibrin-alginate hydrogels enhances cartilage matrix synthesis and chondrocyte proliferation, reinforcing its therapeutic potential in OA management [77,96].

### 4.2. Approaches to cartilage regeneration

Bioengineering integrates engineering and biological principles to create biological replacements for regenerating damaged tissues. Utilizing nanotechnology, biomaterials, stem cells, and signaling biomolecules, advances in biomedical engineering, particularly in 3D bioprinting, have significantly improved cartilage repair. 3D bioprinting is an advanced fabrication technology that enables the precise spatial arrangement of cells, biomaterials, and bioactive molecules to construct functional tissue structures. Unlike traditional scaffold-based methods, 3D bioprinting allows for controlled deposition of bioinks, facilitating the development of biomimetic tissue constructs with improved structural and biological fidelity. This technique enhances the potential for bioidentical tissue engineering by enabling the recreation of complex cartilage architectures essential for OA treatment [97]. Approaches to cartilage regeneration using static and dynamic culture systems and 3D bioprinting technologies are at the forefront of regenerative medicine, offering solutions for cartilage repair and OA. Cartilage regeneration relies on the creation of an environment that can mimic natural cartilage tissue. Both static and dynamic culture systems as shown in Figure 6, which provides the platform for growing cells in a way that supports tissue engineering. The major difference lies in how the environmental stimuli are provided to the cells. 3D bioprinting technology allows precise deposition of cells and biomaterials in three dimensions to create constructs that mimic the structure and function of native cartilage. 3D bioprinting, utilizing techniques like extrusion, inkjet, laser-assisted, and stereolithography as shown in Figure 7, is revolutionizing the creation of complex cartilage structures. The combination of advanced bioprinting techniques with appropriate bioinks offers promising avenues for producing functional, durable cartilage tissues for clinical applications.

**Figure 6.** Conventional approaches for cartilage regeneration.

**Figure 7.** 3D bioprinting approaches for cartilage regeneration.

## 5. Biomaterials based cartilage regeneration and osteoarthritis treatment

Biomaterials serve as essential carriers for delivering gene therapies to OA-affected tissues, facilitating targeted and efficient treatment. The choice of suitable biomaterials is influenced by critical factors such as biocompatibility, biodegradability, and mechanical properties, all of which play a pivotal role in ensuring the effectiveness and accuracy of gene therapy delivery to the intended site. Various biomaterials, including metallic implants, hydrogels, nanoparticles, liposomes, micelles, and dendrimers, have shown significant potential in OA treatment. Their ability to enhance drug stability, facilitate controlled release, and improve cellular uptake makes them valuable tools in regenerative medicine. The importance of these biomaterials in OA therapy is highlighted in Table 2.

**Table 2.** Comparison of biomaterials for OA treatment.

Biomaterials	Roles in OA	Mechanism	Advantages	Disadvantages	Reference
Metallic implants	Provide durable and strong support for joint function; Often used in joint replacement surgeries	Offer long-term support for joint function; Potential for metal ion release into the bloodstream, causing inflammation and tissue damage; Risk of implant loosening or failure over time	Durable and strong, providing long-term support for joint function. Can be custom designed for individual patients. Often used in joint replacement surgeries	Potential for metal ion release into the bloodstream, causing inflammation and tissue damage. Risk of implant loosening or failure over time	[98]
Hydrogels	Simulate the gel-like ECM of joint tissue; ensure sustained and controlled release of therapeutic agents.	Prevent cartilage degradation, stimulate cartilage repair, and inhibit synovial hyperplasia.	Possess a highly hydrated polymeric structure that mimics the ECM	Hydrogels derived from natural polymers have limited mechanical strength and are susceptible to enzymatic degradation; mechanical properties can be improved using synthetic polymers.	[99–102]
Nanoparticles	Enable controlled and site-specific delivery of therapeutic agents; allow deeper penetration into complex joint structures.	Facilitate cartilage regeneration, alleviate inflammation, and provide pain relief.	Ability to pass through cartilage mesh (pore size of 60–200 nm), ensuring sustained drug release within the ECM; can be absorbed by chondrocytes and synoviocytes.	Rapid clearance by the synovial microvascular system; can be enhanced using targeted binding strategies; concerns regarding potential toxicity.	[103,104]
Microparticles	Provide an optimal microenvironment for cell adhesion and proliferation; allow for controlled and prolonged release of therapeutic molecules.	Stimulate cartilage regeneration, reduce inflammation, alleviate synovial hyperplasia, and promote pain relief.	Microparticles smaller than 10 µm are internalized by synovial macrophages and chondrocytes; larger particles (>10 µm) exhibit a slower clearance rate, remaining in the joint longer.	Unable to penetrate the ECM; prolonged retention may increase the risk of toxicity and adverse effects.	[105–108]
Liposomes	Deliver bioactive molecules over an extended period while ensuring localized and targeted drug release.	Encourage tissue repair, modulate chronic inflammation, and support cartilage regeneration.	Capable of encapsulating both hydrophilic and hydrophobic drugs; exhibit excellent biocompatibility as lipids are naturally found in cell membranes; available in a variety of nano- and micro-sizes; function as both a drug delivery system (DDS) and a joint lubricant.	Susceptible to physical instability, which may lead to drug leakage.	[109–112]
Dendrimers and micelles	Ensure sustained and stable release of therapeutic agents; enhance drug solubility and stability.	Inhibit synovial hyperplasia, reduce inflammation, and accelerate cartilage repair.	Nanoscale size allows easy penetration into the ECM; well-controlled physicochemical characteristics (high monodispersity, defined functional groups, and strong cationic charges for cartilage targeting).	Cellular toxicity (hemolytic activity) due to excessive positive primary amine groups; biocompatibility can be improved through polyethylene glycol (PEG) modification.	[113–116]

### 5.1. Metallic implant

Metallic implants are primarily used in orthopedic applications for structural support, such as joint replacements or fracture fixation as shown in Figure 8. Metal elements are an essential component of our human bodies and present in an adequate amount such as Na, Ca, Mg, Zn, Co, Si etc [98]. The two types of biomaterials that are typically used in attempts to decrease osteoporotic fractures are metallic implants and cements. Metallic materials like stainless steels, titanium alloys, and cobalt alloys are used in orthopedic treatments for surgical implants like plates, fixation screws, and artificial joints. These materials have exceptional mechanical properties, making them ideal for load-bearing implants [117]. Cements are used to strengthen the hardware, while titanium implants have a high success rate [118]. The choice of implant composition made with the intention of enhancing osseointegration is a key sign of the clinical success of the device [119]. Ti-based alloy (Ti–6Al–4 V), and many other metals (such as dental amalgam, tantalum, and gold combined with other ‘specialty’ metals) are currently the metal biomaterials that are beneficial in the biomedical area [120].

**Figure 8.** Clinical applications of metallic implants.

Osteosynthesis screws can be increased in diameter and locked osteosynthesis plates can be used for vertebral height restoration. New trochanteric and displaced intracapsular fractures can be created using implants like cannulated screws or expandable spacers [121]. Controlled medication distribution is enabled by metallic and oxide nanoparticles as referred in Table 3, affixed to orthopedic implants and scaffolds, which can respond to stimuli. These nanoparticles can be coated or encapsulated in biodegradable or nonbiodegradable forms, such as poly-lactic acid (PLA), to facilitate targeted therapy and faster bone regeneration. Metal implants can release targeted metal elements into tissues at modest corrosion rates, providing specific biofunctions [142]. A new type of stainless steel, 316 L-Cu, has been developed to replace 316 L used for stents. Copper ions can facilitate intraosseous vascular repair and collagen deposition, benefiting osteogenesis. 317 L-Cu steel promoted osteogenesis, accelerating bone fusion and implant-bone bonding. It also has anti-bacterial properties, making it a suitable choice for developing a novel stainless steel [143].

**Table 3.** Metallic and metallic oxide nanoparticles in studies pertaining to bones.

S. No	Type of nanoparticle	Role	Cells/animal models Used		Outcome	Reference
1	NPs Silver 75 nm	Antibacterial action	Rat model	Reduced bacterial infection, promoting a healthier environment for cartilage healing		[122]
2	NPs of silver, 20–40 nm	Antibacterial activity	Mouse model	Effective in reducing bacterial colonies, aiding in infection control		[123]
3	Silver nanoparticles and tannic acid	More prone to NPs, antibiofilm activity	In vitro biofilm model	Significantly diminished biofilm formation, aiding in better joint health		[124]
4	Gold NPs	Improve micro-CT visibility; strong osteogenic and cytocompatibility properties	Mouse model	Enhanced visibility in imaging; Promoted bone regeneration and better biocompatibility		[125]
5	Gold NPs	Targeted delivery to injured bone tissue	Rat model	Focused treatment leading to better healing outcomes in damaged bone tissues		[126]
6	Gold	Elevated ROS production	In vitro cell culture model	Improved oxidative stress response, promoting an environment conducive to cartilage repair		[127,128]
7	Gold	Antimicrobial properties	Mouse model	Reduced microbial infection, helping maintain joint health		[129]
8	NPs of copper	Antibacterial and antifungal properties; ROS production	Rat model, fungal culture model	Effective in reducing bacterial and fungal presence, fostering a supportive environment for cartilage regeneration		[130–132]
9	Cerium-oxide nanoparticles, Titanium oxide NPs, and Zinc oxide NPs	Antibacterial action	In vitro bacterial culture model	Improved infection control, aiding in better joint and cartilage health		[133]
10	Tantalum	Biocompatibility, low toxicity, and photoacoustic effect	Mouse model of tumors	Enhanced imaging of tumors; Potential for targeted therapy in osteoarthritic conditions		[134]
11	Ta_2_O_5_	High affinity for articular cartilage due to coulombic attraction	In vitro cartilage affinity model	Better integration and repair in cartilage applications		[135]
12	SPIONs	Osteogenic, chondrogenic, and adipogenic differentiation; MRI detection	Bone marrow-derived stem cells (BMSCs) and adipose-derived stem cells (ADSCs)	Improved visualization and tracking of stem cells in joint tissues; Promoted cartilage and bone formation		[136]
13	SPIONs	Reduced adipogenic and osteogenic differentiation with increased concentrations; easier detection of stem cells	hADSCs and BMSCs	Easier detection of stem cells, reduced differentiation and survival with higher SPION concentrations		[137]
14	Zinc-oxide Nanoparticles	Damage to membrane integrity and ROS generation	Bacterial culture model	Improved oxidative stress response and microbial control		[138]
15	Zinc-oxide Nanoparticles	Antimicrobial mechanism via hydrogen peroxide	Bacterial culture model	Enhanced control over microbial presence, promoting a healthier joint environment		[139]
16	Composite of Ag-ZnO	ROS generation and release of Ag^+^ and Zn	In vitro cell culture model	Enhanced microbial control and oxidative stress response, aiding in cartilage repair		[140]
17	Zinc-oxide nanocatalyst	Production of OH^−^, H_2_O_2_, and additional ROS	In vitro cell culture model	Improved oxidative stress response, supporting cartilage health		[141]

### 5.2. Hydrogel

Hydrogels can be engineered with varied three-dimensional architectures, porosities, elastic properties, and mechanical strengths by selecting specific molecular monomer reagents and crosslinking them in aqueous environments using physical or chemical techniques, resulting in insoluble network structures [144]. As biocompatible materials, hydrogels maintain high water retention due to their crosslinked networks, which exhibit complex physical and chemical characteristics. This unique structure allows hydrogels to replicate the extracellular matrix (ECM), fostering a supportive microenvironment for cell viability and tissue regeneration.

**Hyaluronic acid** is a linear polysaccharide and a fundamental component of cartilage ECM, extensively explored for its role in cartilage regeneration and OA treatment [145]. It serves as a lubricant and plays a role in modulating inflammatory responses, cell adhesion, migration, proliferation, differentiation, angiogenesis, and tissue regeneration [146–150]. In clinical practice, HA is commonly administered weekly as a visco supplement to alleviate pain [151]. Non-crosslinked hyaluronic acid (HA) solutions often lack structural stability, resulting in short retention times and limited ability to deliver bioactive agents. To address this issue, HA is chemically modified to form hydrogels, improving its therapeutic potential [152]. While HA-based hydrogels possess mucoadhesive properties, they typically exhibit weak tissue adhesion [153,154]. To enhance retention and effectiveness, various functional adhesive groups such as catechol, methacrylate, aldehyde, tyramine, and o-nitrobenzyl alcohol have been incorporated into HA [155–159]. This modification significantly strengthens HA-based hydrogel adhesion, improving integration between newly formed cartilage and host tissue, thereby enhancing therapeutic outcomes. Chen et al. [160] chemically modified HA by incorporating aldehyde groups and employed photo-crosslinking techniques to create an adhesive hydrogel with stronger adhesion than fibrin glue. In vivo studies confirmed that these HA-based adhesive hydrogels facilitated superior cartilage regeneration and better integration with host tissue than non-adhesive alternatives.

**Alginate**, derived from brown algae or bacteria, is widely used in biomedical applications due to its biocompatibility and easy gelation [147]. However, alginate hydrogels tend to have poor tissue adhesion, requiring chemical modifications to improve their bonding ability [90]. One of the most common modifications involves oxidizing alginate polymer chains to introduce aldehyde groups, enabling crosslinking with amino-containing molecules to form adhesive hydrogels. Since alginate-based hydrogels have great potential for cell and gene delivery [74,147], they are also employed in cartilage regeneration and OA treatment. Kreller et al. [148] developed a 3D-printed hydrogel using oxidized alginate and gelatin (ADA-GEL) for cartilage tissue engineering. ADA-GEL exhibited high structural stability, allowing it to be printed into complex scaffolds that encapsulate cells while mimicking the hierarchical structure of native cartilage, making it a promising approach for OA therapy. Besides natural crosslinking with amino-containing biomolecules, synthetic polymers with amino groups can also be linked to aldehyde-modified alginate. Yan et al. [161] designed injectable adhesive hydrogels by crosslinking aldehyde-modified alginate with hydrazide-modified poly (L-glutamic acid). By modifying solid content and oxidation levels, these hydrogels displayed adjustable mechanical properties and degradation rates. Compared to direct chondrocyte injections, chondrocyte-loaded adhesive hydrogels facilitated the formation of cartilage-like tissue, better maintaining its shape and structural integrity.

**Chitosan**, obtained through the partial deacetylation of chitin [162], is widely recognized for its versatility, biocompatibility, biodegradability, and antimicrobial properties, making it a key material in tissue engineering and regenerative medicine. As illustrated in Figure 9, chitosan scaffolds play a crucial role in cartilage regeneration, supporting tissue repair and structural integrity. Additionally, chitosan exhibits unique biological properties, including tissue adhesion, antioxidant activity, antibacterial effects, and anticancer potential, making it the only naturally occurring polysaccharide with a positive charge [81]. Beyond these intrinsic properties, chitosan can be chemically modified to expand its applications, resulting in derivatives such as thiolated chitosan and hydroxyalkyl chitosan. Scognamiglio et al. [163] synthesized a lactose-modified chitosan hydrogel (CTL-hydrogel) using boric acid crosslinking. This chitosan-based adhesive hydrogel exhibited greater stability than traditional HA solutions, offering longer-lasting visco-supplementation for OA treatment. Additionally, lactose-modified chitosan displayed antioxidant properties, making CTL-hydrogel an effective reactive oxygen species (ROS) scavenger, further enhancing its therapeutic potential for OA therapy.

**Figure 9.** Development of chitosan based bioproducts in the treatment of OA.

**Chondroitin sulfate** is a sulfated glycosaminoglycan (GAG) consisting of N-acetylgalactosamine and glucuronic acid, playing a crucial role in the cartilage ECM. It is known for its anti-inflammatory, antioxidative, and anti-apoptotic properties, while also stimulating the production of hyaluronan, collagen, and glucosamine. Additionally, CS helps prevent ECM degradation and has long been used as a dietary supplement for OA to reduce pain and promote cartilage regeneration. Despite having some tissue adhesion capabilities due to hydroxyl, carboxyl, and amide groups, its adhesion strength is relatively low [164]. To improve its tissue-binding properties, CS is chemically modified with functional adhesive groups such as thiol and aldehyde.

**Gelatin**, a water-soluble natural polymer, is derived from collagen hydrolysis. Collagen plays an important role in joint protection by mobilizing T regulatory cells and encouraging the production of anti-inflammatory cytokines [165,166]. Collagen-based hydrogels have been investigated for their potential in repairing OA-related cartilage defects due to their ability to stimulate the expression of essential ECM molecules such as Agc1, Col2α1-IIa, and SOX9, which contribute to cartilage formation [167]. However, these hydrogels lack mechanical strength and degrade quickly [168]. Furthermore, due to collagen’s low water solubility and thermostability, the complex chemical modification process has restricted its use in developing adhesive hydrogels for OA treatment [169]. Gelatin, in contrast, has gained attention in tissue regeneration due to its excellent biocompatibility, biodegradability, low immunogenicity, high water solubility, and ease of modification [170]. Gelatin-based materials also adhere to tissues through electrostatic interactions, mediated by amino and carboxyl groups. Zhang et al. [171] designed gelatin microcryogels to deliver mesenchymal stem cells (MSCs), significantly improving MSC retention in the knee joints of mice when compared to direct MSC injections. However, non-covalently crosslinked gelatin alone has insufficient mechanical strength. To overcome this, gelatin is often combined with aldehyde-containing materials to create adhesive hydrogels for OA therapy [161,172]. Moreover, gelatin’s amino and carboxyl groups can be chemically modified to further enhance its adhesive properties. Lim et al. [173] modified gelatin using tyramine and methacryloyl to develop a highly adhesive hydrogel through photo-crosslinking, which improved adhesion strength by 15-fold compared to methacrylated gelatin (GelMA). The hydrogel encapsulating articular chondroprogenitor cells demonstrated an increased collagen type-II/I ratio, indicative of chondrogenic differentiation.

**Mussel adhesive proteins** (MAPs), secreted by marine mussels, enable strong adhesion to various surfaces in turbulent aquatic environments through DOPA-mediated interfacial bonding. These proteins have been widely studied for their applications in wound healing and cell adhesion [174,175]. Stem cell therapy has been explored for cartilage regeneration in OA treatment for over two decades, but challenges such as low cell viability and unintended cell dispersion remain. Studies have shown that adipose-derived stem cells (ASCs) immobilized using MAPs exhibit improved retention on chondral defects compared to fibrin glue-secured ASCs. Ko et al. [176] used MAP-based adhesives to firmly attach human ASCs with enhanced chondrogenic potential to damaged cartilage sites, extending their survival and promoting differentiation into chondrocytes. This prolonged stem cell retention may enhance therapeutic effectiveness by ensuring sustained paracrine signaling and improved engraftment.

**Fibrin glue** is a two-component topical hemostatic agent and tissue adhesive, consisting of fibrinogen and thrombin. Commercially available since the late 1970s, it is FDA-approved for multiple applications, including hemostasis, securing burn wound grafts, and sealing colon defects. Fibrin networks resemble natural ECM, providing excellent biocompatibility, biodegradability, and cell-binding properties [84]. Clinical research suggests that implanting MSCs using fibrin glue enhances OA treatment efficacy compared to MSC implantation alone, as determined by the International Cartilage Repair Society grading system [177]. However, since fibrin glue components are derived from human or animal blood, there is a potential risk of serological disease transmission.

### 5.3. Nano scale particles

Nanoparticles have emerged as a versatile and efficient strategy for delivering small molecules in OA therapy. These nanocarriers enable precise encapsulation and controlled release of therapeutic agents, improving treatment accuracy and efficacy [178]. Their unique physicochemical properties, including size, surface charge, and hydrophobicity, can be tailored to enhance their performance and maximize therapeutic benefits. Among various polymeric materials used for fabricating nanoparticles, poly(lactic-co-glycolic acid) (PLGA) is one of the most extensively studied due to its biocompatibility and biodegradability, making it well-suited for biomedical applications [179]. PLGA nanoparticles have demonstrated great potential in targeted drug delivery for OA management. For instance, Kim et al. [180] designed rebamipide-loaded nanoparticles using methoxy poly (ethylene glycol)-b-poly(D, L-lactide) (mPEG-PDLLA) and PLGA polymers to achieve sustained drug release. In in vitro studies, these nanoparticles effectively downregulated mRNA levels of pro-inflammatory mediators, including IL-1β, IL-6, TNF-α, MMP-3, MMP-13, and cyclooxygenase-2, in a dose-dependent manner. Additionally, in vivo experiments demonstrated that intra-articular administration of rebamipide-loaded nanoparticles resulted in the greatest reduction in inflammatory mediator mRNA levels compared to other treatment methods. Macroscopic, radiographic, and histological assessments further confirmed that these nanoparticles effectively inhibited cartilage degeneration, outperforming both oral rebamipide administration and rebamipide solution injections. These findings highlight that delivering rebamipide through intra-articular injections, particularly when encapsulated in PLGA nanoparticles, helps reduce inflammation, prevent cartilage breakdown, and slow OA progression.

Beyond delivering anti-inflammatory drugs, PLGA nanoparticles have been engineered to enhance chondrogenesis and cartilage repair. One notable example is p66shc, a protein highly expressed in OA cartilage, which plays a key role in disease progression. The use of p66shc small interfering RNA (siRNA)-loaded PLGA nanoparticles allows for sustained release, prolonging its presence within the joint microenvironment. In vivo studies revealed that p66shc inhibition via siRNA-loaded PLGA nanoparticles significantly reduced pain behavior, minimized cartilage degradation, and suppressed inflammatory cytokine production in OA rat knee joints. These findings suggest that p66shc siRNA-loaded PLGA nanoparticles may be an effective therapeutic strategy for OA management [181]. In addition to their ability to deliver targeted therapies, polymeric nanoparticles offer several key advantages for OA treatment. Their nanoscale size allows for efficient penetration into dense joint spaces, ensuring precise delivery to affected tissues. Additionally, their controlled-release capabilities enable a sustained therapeutic effect, reducing dosing frequency while optimizing drug bioavailability. Furthermore, modifications to nanoparticle surface properties can enhance their stability, cellular uptake, and interaction with joint tissues, further improving overall treatment efficacy.

### 5.4. Liposomes

Liposomes, which can be designed in tunable micro- or nano-sized structures, offer the ability to encapsulate both hydrophilic and hydrophobic drugs within their aqueous core and phospholipid bilayer, respectively. Additionally, due to the lubricating properties of phospholipids (PLs), liposomes can serve a dual function by enhancing joint lubrication while delivering therapeutic agents. For instance, distearoylphosphatidylcholine (DSPC) liposomes enabled the controlled release of glucosamine (GAS) for a duration of up to 14 days, effectively reducing the coefficient of friction (CoF) to 0.03, which is significantly lower compared to water (0.3).This dual effect improved both drug retention and lubrication. Although DSPC-GAS liposomes demonstrated only slightly better results than free GAS, they effectively reduced inflammatory and catabolic markers in TNF-α-stimulated chondrocytes, including IL-1β, IL-6, and MMP1 mRNA. At the same time, they enhanced mRNA expression of aggrecan and type II collagen (COL II) within 24 hours due to the controlled release of GAS from the delivery system. These findings highlight the chondroprotective properties of liposomal formulations [182]. Yeh et al. demonstrated that incorporating specific therapeutic agents into liposomes enhanced drug uptake in bone tissue [183]. Frisbie et al. investigated the effectiveness of diclofenac liposomal cream (DLC) in horses with OA and found that treatment led to a notable decrease in radial wrist sclerosis and cartilage degradation. The study also revealed a notable increase in glycosaminoglycan content within the articular cartilage while simultaneously lowering prostaglandin E2 (PGE2) levels. Furthermore, no treatment-related side effects were reported, confirming the safety and therapeutic potential of liposomal formulations for OA management [184]. Furthermore, Sivan et al. explored the effectiveness of liposomes formulated with various phosphatidylcholines (PCs) as high-performance cartilage biolubricants. One of the key advantages of liposomes is their ability to protect encapsulated drugs from metabolic degradation, thereby extending their half-life. By modifying their size or surface properties, often through polyethylene glycol (PEG) conjugation, liposomes can achieve prolonged circulation times. Moreover, specifically engineered liposomes can be designed to target particular cells or anatomical locations such as the cartilage surface, synovial membrane, or articular space [185]. Compared to free drugs, liposomal formulations have been shown to significantly reduce cytotoxicity and adverse effects, further underscoring their potential in OA therapy.

### 5.5. Micelles and dendrimers

Micelles, characterized by their core – shell structure, have emerged as highly promising carriers due to their excellent biocompatibility and controlled drug release properties. Matsuzaki et al. examined the potential of rapamycin-loaded micelles for OA therapy through intra-articular (IA) injection [186]. Compared to gelatin hydrogels alone, rapamycin-micelles exhibited long-lasting therapeutic effects, maintaining significantly lower OA scores over time. Similarly, Zhang et al. developed amphiphilic micelles to encapsulate indomethacin, a commonly used nonsteroidal anti-inflammatory drug (NSAID). Polymeric micelles have emerged as a versatile and effective platform for delivering small molecules in OA treatment [114]. These self-assembling nanostructures, composed of amphiphilic polymers, enhance the solubility, stability, and controlled release of hydrophobic drugs, making them highly suitable for OA therapy. A distinctive feature of polymeric micelles is their ability to encapsulate hydrophobic drugs within their core structure. When dispersed in an aqueous medium, the hydrophobic segments of amphiphilic polymers cluster together to form a central core, while the hydrophilic segments create a protective outer shell, stabilizing the micelle structure. This unique configuration enhances drug solubility, while also protecting the encapsulated drugs from enzymatic degradation and premature release.

Among various polymeric micelles, polyethylene glycol (PEG)-based micelles have attracted significant interest for their applications in OA drug delivery [187]. PEG-poly(lactic acid) (PEG-PLA) micelles combine PEG’s hydrophilic properties with PLA’s biodegradability, providing an efficient drug delivery platform. The PEG shell extends micelle stability and circulation time, while the PLA core serves as a carrier for small molecules. Dexamethasone, a potent anti-inflammatory drug, has been successfully encapsulated in PEG-PLA micelles, offering localized and sustained release to reduce inflammation and pain in OA patients. Similarly, PEG-poly(caprolactone) (PEG-PCL) micelles have demonstrated strong potential for OA therapy [115]. These micelles combine the biocompatibility and stability of PEG with the high drug-loading capacity and biodegradability of poly(caprolactone) (PCL), forming an effective drug delivery system. Key anti-inflammatory molecules such as 9-aminoacridine (9AA) and caffeic acid (CA), which contribute to cartilage regeneration, have been successfully incorporated into PEG-PCL nanomicelles [116]. These nanomicelles shield 9AA and CA from enzymatic degradation, enabling a controlled and sustained release, ensuring prolonged therapeutic action within the joint environment.

Dendrimers, derived from the Greek word *dendron*, meaning ‘tree,’ feature a highly branched three-dimensional (3D) architecture comprising a core, an interior, and a shell. These nanocarriers are designed to encapsulate and dissolve hydrophobic drugs within their interior structure. Due to their water solubility, polyvalent nature, and uniform nanoscale structure, dendrimers can efficiently penetrate biological barriers and enable controlled drug delivery. Their therapeutic potential in OA treatment has been widely explored. Research has demonstrated that polyamidoamine (PAMAM) dendrimers loaded with indomethacin can selectively target inflammatory sites in arthritic rat models [185]. Hu et al. [188] investigated the use of PEGylated PAMAM dendrimers as carriers for kartogenin (KGN), a small molecule known to stimulate chondrogenesis. Two types of KGN-loaded dendrimers were developed: one where KGN was conjugated to the PAMAM surface (PPK) and another where KGN was linked to the PEG end group (KPP). Both formulations had a diameter of less than 40 nm. After intra-articular (IA) injection into healthy and OA-affected knee joints, cyanine 7-PEG-PAMAM signals were detectable for up to 21 days in rats, whereas free Cy7 signals disappeared within 24 hours. Importantly, cells treated with KPP displayed the highest expression of chondrogenic markers, suggesting that the enhanced therapeutic effects of KGN were attributed to the prolonged retention of dendrimers within the joint cavity.

## 6. CRISPR/Cas9 in osteoarthritis and their limitations

The CRISPR/Cas system offers an advanced tool for genome editing for the treatment of OA and other degenerative joint conditions. The term ‘clustered regularly interspaced short palindromic repeats,’ which was first identified during research on prokaryotes’ adaptive immune system, is abbreviated as CRISPR [187]. Its mechanism, which is similar to the memory cells found in the human immune system, is regarded to be a helpful way used by bacteria and archaea to remember knowledge about phage viruses and then destroy them on repeated contacts. The CRISPR system enables precise modifications to be made at specific genomic sites in both prokaryotes and eukaryotes, including deletions, insertions, substitutions, and other alterations, when combined with other proteins, particularly endogenously produced enzymes like Cas in prokaryotic cells.

A synthetic guide RNA was created to enhance CRISPR-mediated genome editing efficiency. This RNA facilitates Cas9 endonuclease cleavage by hybridizing with target DNA [189]. The protospacer adjacent motif (PAM) is needed for Cas9 protein binding. By using endogenous promoter sequences, like CRISPR, in anti-inflammatory therapies like rheumatoid arthritis, genome editing technologies have the potential to transform cell-based anti-cytokine therapy. In a recent study, using the CRISPR-Cas9 genome editing technique, a stem cell system that targets cytokines and is self-regulating in mouse induced pluripotent stem cells (iPSCs) was developed [190]. The potential for induced pluripotent stem cells (iPSCs) to differentiate into various cell types in the future. The primary goal of these modified cells was to transcribe soluble receptors for TNF - α (sTNFR1), interleukin-1 receptor antagonist (IL1Ra), or luciferase (used as a control) using the built-in promoter for macrophage chemoattractant protein-1 (Ccl2). This was carried out under feedback control. Considering the significance of the Ccl2 and NF-kB signaling pathways in the development and progression of pain and structural degeneration in OA, using this could be a viable therapeutic approach [191].

Researchers Seidl et al. used CRISPR gene editing techniques to increase collagen type 2 expression in human articular chondrocytes, a key component in OA treatment. They transfected the MMP13 gene into HACs, reducing MMP13 protein levels and enzymatic activity. The study found that genetic changes at the MMP13 locus resulted in a 50% efficiency rate. The cells genetically engineered to express MMP13 produced more collagen type 2, crucial for maintaining cartilage structural integrity and joint functionality. The findings suggest that CRISPR gene editing could be a viable treatment option for OA [192].

Mutations in mitochondrial genes are linked to OA, and genome editing techniques can be used to fix these mutations and restore healthy mitochondrial DNA (mtDNA). This approach aims to promote mitochondrial function while reducing OA symptoms. Researchers have used CRISPR/Cas9 to target Cox1 and Cox3 in mtDNA, suppressing cell growth and modifying the potential of the mitochondrial membrane. However, modifying mtDNA using CRISPR/Cas9 is challenging due to the double-layered mitochondrial membrane. Researchers hope to repair the damage caused by the MT-TK mutation in mt-tRNALys, potentially helping cure mitochondrial diseases caused by anomalies in mtDNA [193].

### 6.1. The molecular targets of CRISPR/Cas9 in the context of therapeutic intervention for osteoarthritis

The potential of cell therapy in the treatment of OA is considerable; nevertheless, the efficacy of repairing articular cartilage by stem cell-based approaches might be impeded by the presence of inflammation. To proficiently administer OA, it is necessary to evaluate and focus on inflammation and its correlated components. Several research institutions are actively exploring the potential of CRISPR/Cas9 technology for osteoarthritis (OA) treatment. This gene-editing tool is extensively utilized in the field of genetic engineering [190]. IL-1β, a pro-inflammatory cytokine, is predominantly produced by neutrophils and plays a crucial role in inflammatory processes. The overexpression of IL-1β results in the upregulation of many genes that are related with OA as well as other cytokines, such as TNF-α. Presently, the therapy of OA mostly centers on the inhibition of TNF-α. Nevertheless, the efficacy of these therapies is constrained because of the involvement of TNF-α in several physiological processes. It is noteworthy that the exposure to TNF-α results in heightened production of IL-1β in human articular cartilage (hAC) [194,195]. The IL-1β cytokine receptor (IL1-R1) was successfully inhibited in human articular chondrocytes (hACs) by Karlsen et al. (2016) to investigate its impact on inflammation and hACs’ ability to redifferentiate after being exposed to IL-1β [196].

A puromycin-resistance gene was simultaneously introduced, and the IL1-R1 receptor gene was specifically disrupted using the CRISPR/Cas9 system on human articular chondrocytes (HACs) isolated from cartilage tissue. Spotting and isolating cells that have the necessary knockout phenotype has been made easier with the help of genetic editing techniques. Subsequently, the knockout cell colonies were subjected to exposure with recombinant IL-1β and TNF-α in order to evaluate their respective reactions [194]. Certain findings demonstrated that the introduction of recombinant IL-1β resulted in a notable escalation of inflammation within the control group, aligning with the anticipated outcome. Nevertheless, within the experimental group in which the IL1-R1 gene was eliminated, the administration of recombinant IL-1β failed to elicit any observable indications of inflammation. This suggests that blocking IL1-R1 in vitro in articular cartilage cells before reintroducing them into the body could potentially enhance the outcomes of cell therapy [190].

In contemporary scientific pursuits, there has been a notable focus on the manipulation of cellular senescence using gene-editing techniques. The study conducted by Ren et al. provided evidence of the significant influence of altering CBX4 in mitigating cellular senescence, hence providing beneficial outcomes in the context of OA [197]. The transcriptional co-activator known as YAP has the capability to modulate the activity of the FOXD1 transcription factor. Based on contemporary study findings, the activation of YAP can increase the expression of FOXD1, therefore presenting a viable approach to mitigate OA through the reduction of cellular senescence. Subsequent investigations pertaining to the modification of connexin 43 have shown that the attenuation of cellular senescence has promise in augmenting the regeneration capacities of cells and enhancing the quality of tissues within the framework of OA [190,198]. The use of CRISPR/Cas9 technology has enabled the discovery of additional targets that can be potentially targeted for therapeutic treatments. Using CRISPR/Cas9 technology to disrupt the hyaluronan synthase 2 (HAS2) gene in rat chondrocytes demonstrated how important the glycosaminoglycan hyaluronan is for the preservation of aggrecan, a proteoglycan that is essential for preserving the articular cartilage’s ability to function properly. Consequently, the CRISPR/Cas9 system can offer important insights into the molecular processes necessary for preserving the health of joint tissue which showed a promising therapeutic intervention [199,200].

## 6.2. CRISPR/Cas9 system and biomaterial based gene delivery

Hydrogels have gained recognition as a versatile platform for gene delivery in OA, allowing for multiple administration methods, including direct intra-articular injection or implantable hydrogel scaffolds that provide sustained release of gene therapy. The success of hydrogel-based gene delivery is influenced by several critical factors, such as biocompatibility, biodegradability, mechanical strength, and the ability to encapsulate and efficiently release therapeutic genes [201–205]. Among the different hydrogel systems investigated for gene therapy in OA, chitosan-based hydrogels have demonstrated significant therapeutic potential. Chitosan, a biodegradable polysaccharide derived from chitin found in crustacean exoskeletons, is widely recognized for its excellent biocompatibility and ability to deliver nucleic acids effectively [206]. These hydrogels can undergo chemical modifications to improve their ability to target specific tissues. Man et al. designed a hybrid scaffold consisting of chitosan hydrogel and demineralized bone matrix (DBM) to promote cartilage regeneration in a rabbit model [207,208]. Both in vitro and in vivo studies demonstrated that allogenic chondrocyte transplantation using the chitosan – DBM scaffold effectively repaired cartilage damage in a single-step procedure. Another study demonstrated the potential of hyaluronic acid hydrogels for gene therapy by successfully delivering the CRISPR/Cas9 system into mesenchymal stem cells in vitro. This approach enabled precise gene editing, promoting cartilage regeneration. Additionally, other hydrogel-based gene delivery platforms, such as hyaluronic acid, alginate, and fibrin-based hydrogels, have been explored for OA treatment [74,209]. Preclinical studies have shown promising outcomes for these gene delivery systems, demonstrating their ability to effectively encapsulate and transport therapeutic genes. However, additional research is necessary to thoroughly assess their safety, efficacy, and long-term clinical viability.

A recent breakthrough involved the use of PAsp (MTAS-NLS-co-DMH), a cationic polymer complex, to create nanoparticles by binding them with plasmids encoding the CRISPR activation (CRISPRa) system, which were subsequently transfected into MC3T3-E1 cells. Once inside the cells, the pH-sensitive dimethyl-histidine (DMH) moiety triggered lysosomal rupture, allowing the nanoparticles to escape into the cytoplasm through the proton sponge effect. Following this, the nuclear-localizing peptide NLS-MTAS directed the plasmid into the nucleus, enabling the expression of mRNAs encoding the dCas9 protein and sgRNA. To create an injectable format for the CRISPRa-engineered MC3T3-E1 cells, researchers synthesized a dual cross-linked hyaluronic acid hydrogel using Schiff-base and azide – alkyne cycloaddition reactions. This innovative system utilized a slow-reacting aldehyde-oxyamine conjugation combined with a rapid N3-DBCO (dibenzocyclooctyne-succinimide ester) conjugation, ensuring high cellular uptake efficiency and controlled cell release. As anticipated, the scaffold significantly improved calvarial bone healing by enhancing both angiogenesis and osteogenesis in vivo. The simultaneous activation of TGF-β1 and VEGF-A genes resulted in greater bone formation compared to the activation of a single gene [210]. These findings underscore the tremendous potential of hydrogel-based gene therapy in advancing OA treatment.

### 6.3. PAM recognition of CRISPR

The requirement of a protospacer adjacent motif (PAM) sequence poses a significant limitation when utilizing SpCas9-based systems for OA therapy, as SpCas9 specifically recognizes the PAM sequence *5’-NGG-3“* [211]. To overcome this constraint and expand the targeting range, researchers have explored various Cas9 orthologs that recognize different PAM sequences. Several alternative Cas9 variants have been explored, including SaCas9 (5”-NNGRRT-3“), StCas9 (*Streptococcus thermophilus* Cas9, 5”-NAG-3“), SauriCas9 (*Staphylococcus auricularis* Cas9, 5”-NNGG-3“), CjCas9 (5”-NNNNRYAC-3“), and NmeCas9 (*Neisseria meningitidis* Cas9, 5”-NNNNGATT-3’), each recognizing distinct protospacer adjacent motifs (PAMs) [212–215]. In addition to exploring orthologous Cas9 variants, researchers have engineered SpCas9 through directed evolution and site-specific mutations to reduce its strict PAM dependency.

Phage-assisted continuous evolution (PACE) to modify SpCas9, leading to the discovery of mutants capable of recognizing the NRNH PAM sequence. Meanwhile, through high-throughput analysis and rational design, researchers have developed SpG (5’-NG-3“) and SpRY (5”-NRN-3“ > 5”-NYN-3’) variants, which exhibit expanded PAM recognition capabilities [216]. These variants have already been effectively utilized in genome editing in rice, demonstrating high efficiency in modifying multiple genomic sites. Additionally, base editors and prime editors (PEs) derived from SpRY have been developed, enabling precise DNA modifications without introducing double-strand breaks (DSBs) while maintaining broad compatibility [217–220].

Recently, PESpRY was utilized to correct mutations associated with retinitis pigmentosa (RP). In this study, RP mice carrying PDE6B gene mutations were treated with a dual adeno-associated virus (AAV) vector system delivering the PE-SpRY tool. The treatment successfully restored functional PDE6B protein expression, rescued neural photoreceptor cells, and significantly improved the visual function of the affected mice [221]. These advancements have significantly broadened the scope of CRISPR/Cas technology, enabling greater flexibility in genome targeting. Notably, SpRY has shown the capability to edit nearly all genomic regions without being restricted by PAM sequences. However, its efficiency in recognizing 5’-NYN-3’ PAM sites remains suboptimal, emphasizing the need for further refinement or the development of new Cas9 orthologs to completely eliminate PAM limitations. Overcoming this challenge would pave the way for more adaptable and precise genome-editing approaches in OA therapy [222].

### 6.4. Off-target effects

A major challenge in genome editing technologies is the occurrence of genome-wide off-target effects, which result in unintended modifications in non-targeted genomic regions. To improve the specificity of SpCas9, researchers have engineered several high-fidelity variants, such as eSpCas9, SpCas9-HF1, and HypaCas9, using rational protein design to effectively minimize off-target activity. However, these modifications have also resulted in decreased cleavage kinetics and reduced editing efficiency [223,224]. To maintain on-target activity while minimizing off-target effects, further improvements can be achieved through targeted evolution or advanced rational design. Furthermore, discovering and analyzing new CRISPR/Cas systems from natural sources could lead to the development of advanced genome-editing tools with enhanced precision for targeting OA-associated genes.

Base editors also exhibit off-target effects, which can be categorized as Cas-dependent and Cas-independent. Cas-dependent off-target effects arise from the nonspecific binding of Cas proteins, where high-fidelity Cas9 variants such as eSpCas9, SpCas9-HF1, and HypaCas9 improve specificity by reducing mismatch tolerance in single-guide RNA (sgRNA). Alternative approaches, such as sgRNA truncation and circularly permuted Cas9 architectures, have shown promising results in reducing Cas9-dependent off-target effects [225]. On the other hand, Cas-independent off-target effects result from the random binding of deaminases to either DNA (as seen in cytidine base editors, CBEs) or RNA (affecting both CBEs and adenosine base editors, ABEs). Several cytidine deaminase variants have been engineered to reduce Cas-independent DNA off-target activity, including AALN-BE4, YE1 rAPOBEC1-BE, cA3A-BE3, PpAPOBEC1, RrA3F, AmAPOBEC1, SsAPOBEC3B, A3Bctd-VHM-BE3, and A3Bctd-KKR-BE3 [226–231]. Likewise, specific variants have been designed to minimize Cas-independent RNA off-target activity, such as SECURE-BE3, YE1 rAPOBEC1, cA3A-BE3, PpAPOBEC1, RrA3F, AmAPOBEC1, and SsAPOBEC3B [227,228,230,232]. In adenosine base editors, engineered variants like ABE7.10 (F148W), ABEmaxAW/QW, SECURE-ABE, and ABE8e (V106W) have demonstrated improvements in reducing Cas-independent RNA off-target activity [233,234]. Further modifications to ABE8e led to the development of ABE9, which narrows the editing window while significantly reducing off-target activity in both RNA and Cas9-independent DNA editing [235].

Recent studies have also highlighted potential concerns with RNA-editing tools. Expressing LwaCas13a or PspCas13b in zebrafish embryos has been linked to toxic effects, raising safety considerations for their broader application [236]. As interest in RNA editing continues to grow, newly discovered Cas13 variants, such as Cas13X (775 amino acids) and Cas13Y (790 amino acids), have emerged from the class 2 type VI CRISPR system. These newly identified enzymes are notably smaller than existing Cas13 proteins (~1100 amino acids) and have demonstrated efficient functionality in mammalian cells [237]. However, their off-target collateral activity has not yet been fully assessed. To mitigate concerns related to collateral cleavage by Cas13 enzymes, researchers have developed engineered variants, including hfCas13d and hfCas13×. These modified enzymes preserve on-target RNA degradation while significantly minimizing collateral effects, enhancing the safety of RNA editing and expanding its potential applications [238]. Overall, advancements in genome and RNA editing technologies are continuously refining precision while minimizing unintended modifications. Continued research and optimization of these tools will be essential for ensuring their safe and effective application in OA therapy and other genetic disorders.

## 7. Challenges and future direction

### 7.1. Challenges in biomaterial-based OA therapy

Despite the promising advancements in hydrogel-based and nanotechnology-boosted biomaterials for OA treatment, several challenges hinder their widespread clinical application. These challenges primarily revolve around drug delivery, biocompatibility, mechanical properties, targeted penetration, and regulatory hurdles. One of the significant obstacles is optimizing drug concentration and retention time within hydrogels. While hydrogels offer sustained drug release at the OA site, rapid drug loss due to synovial fluid turnover and joint movement limits their therapeutic efficacy. This necessitates repeated intra-articular injections, which are not only invasive but may also induce joint inflammation, reducing patient compliance. Achieving an ideal hydrogel system that maximizes drug retention while minimizing injection frequency remains an ongoing challenge in biomaterials research.

Another major issue is the mechanical property limitations of hydrogels. Although these biomaterials mimic the ECM of cartilage, traditional hydrogels often lack the required mechanical strength to endure continuous joint loading and compression forces. The mismatch between hydrogel properties and native cartilage restricts their durability and overall functionality in vivo. Thus, enhancing hydrogel strength while maintaining their biocompatibility is a crucial aspect of research. Alongside mechanical considerations, biocompatibility and immune response risks also pose significant challenges. Exogenous stem cells incorporated into hydrogels show promise for cartilage regeneration; however, immune rejection remains a concern. While strategies inducing endogenous stem cell proliferation appear safer, the scarcity of these cells makes achieving adequate regeneration difficult. Additionally, nanoparticles used in drug delivery must ensure safety, avoiding toxicity or unintended accumulation in non-target tissues, which could lead to adverse systemic effects.

Efficiently directing nanoparticles and hydrogels to the affected cartilage while minimizing impact on surrounding tissues is another key challenge. Given that cartilage is avascular, targeted drug delivery remains complex. Furthermore, the extracellular matrix structure of cartilage acts as a natural barrier, hindering the penetration of therapeutic agents. The multifaceted nature of OA, which involves synovial inflammation, subchondral bone changes, and progressive cartilage degradation, further complicates effective targeting. Overcoming these hurdles requires the development of advanced targeting mechanisms, including bioactive surface modifications and smart delivery systems capable of responding to OA-specific microenvironments.

Beyond these biological and mechanical challenges, regulatory and clinical translation barriers also limit the adoption of hydrogel and nanotechnology-based treatments. While many of these therapies have demonstrated success in preclinical studies, only a few have progressed to clinical trials. The regulatory approval process for biomaterials, particularly nanotechnology-enhanced therapeutics, is highly stringent, requiring extensive biocompatibility and efficacy evaluations. Issues such as potential toxicity, immunogenicity, and long-term stability must be rigorously addressed before these therapies can be widely adopted in clinical settings. Establishing standardized testing protocols and frameworks specific to these innovative materials is critical to facilitating their clinical translation. Overcoming these challenges through interdisciplinary collaborations and continued research will be key to realizing the full potential of hydrogels and nanotechnology in revolutionizing OA treatment.

### 7.2. Future directions in OA treatment with biomaterials

To enhance hydrogel-based drug delivery, researchers are exploring advanced modifications, including novel cross-linking techniques, bioadhesive materials, and stimuli-responsive elements. Smart hydrogels capable of responding to pH, temperature, or enzymatic activity can release drugs in a more controlled manner, aligning with the progression of OA. Additionally, hybrid hydrogels that integrate natural and synthetic polymers may improve mechanical properties while maintaining biocompatibility, ensuring both durability and therapeutic efficacy. In parallel, nanotechnology is being integrated into hydrogel systems to improve drug retention and targeted delivery. Functionalizing nanoparticles with surface ligands that bind to specific cartilage biomarkers enhances precision in drug targeting. The use of nanocarriers, such as lipid-based or polymeric nanoparticles, further enhances drug solubility, bioavailability, and controlled release. Additionally, microneedle technology offers a promising alternative to traditional intra-articular injections, allowing for minimally invasive and more efficient drug delivery to the joint.

Advancements in 3D bioprinting technology are revolutionizing OA treatment by enabling the customization of hydrogel structures tailored to individual patient needs. By incorporating patient-specific stem cells and growth factors, 3D-printed hydrogels offer a personalized approach to cartilage regeneration. Furthermore, microfluidic technology is being explored to engineer hydrogel particles with precise size and structure, optimizing their integration within the cartilage matrix. Beyond standalone hydrogel therapies, combination treatments are emerging as a powerful strategy to enhance therapeutic outcomes. By integrating hydrogel-based approaches with other cutting-edge therapies, such as gene editing (CRISPR/Cas9) and regenerative medicine, long-term solutions for OA may be achieved. For instance, hydrogels loaded with chondrogenic growth factors and genetically modified stem cells could significantly enhance cartilage repair while mitigating inflammation. Moreover, bioactive coatings on implants combined with hydrogel-based drug delivery systems may further improve post-surgical outcomes in OA patients.

Addressing the biomechanical limitations of traditional hydrogels is another critical area of research. The development of hydrogels reinforced with nanofibers, self-healing polymers, and nanoparticles like graphene oxide or silica can enhance mechanical strength and resilience. Injectable hydrogels with immediate gelation capabilities may improve integration into the joint environment, while bioinspired superlubricating hydrogels that mimic natural synovial lubrication could reduce friction between cartilage surfaces, thereby improving joint function. Despite these promising advancements, clinical translation remains a major hurdle. Establishing standardized testing protocols and regulatory frameworks tailored to hydrogel and nanotechnology-based OA treatments is essential for accelerating their adoption. Collaboration between material scientists, clinicians, and regulatory authorities will be crucial in streamlining the approval process. Additionally, conducting long-term safety studies and large-scale clinical trials is necessary to validate the efficacy and safety of these innovative therapies, ultimately paving the way for their widespread clinical implementation.

## 8. Conclusion

OA formation is believed to have a significant hereditary component, with studies indicating that at least 30% of the risk of developing the condition is genetically determined. Gaining insights into these genetic factors could lead to the development of more precise and effective treatments. In this regard, future adhesive hydrogel-based therapies should be engineered to provide strong integration for mechanical stability and optimized additive distribution, while also enabling adjustable adhesion between implants and cartilage tissue under diverse conditions. Additionally, these hydrogels should support biological activities through functional components or additives, enhancing their therapeutic impact. Advancements in hydrogel and nanotechnology-based therapies present a promising frontier in OA treatment by offering improved drug delivery, enhanced tissue regeneration, and minimally invasive application. These innovations address the limitations of conventional treatments; however, challenges such as limited drug retention, mechanical deficiencies, immune response risks, and regulatory barriers must be overcome for successful clinical implementation. Future research must focus on developing smart, biocompatible hydrogels with enhanced mechanical properties, integrating nanotechnology for targeted drug delivery, and leveraging 3D bioprinting for personalized OA treatment. Furthermore, combining hydrogel-based therapies with regenerative medicine, gene editing, and bioactive coatings on implants could provide comprehensive solutions for cartilage repair. While clinical translation remains a significant hurdle, ongoing advancements in biomaterials science, bioengineering, and interdisciplinary collaborations will drive the development of more effective, long-term OA therapies. Addressing these challenges and exploring innovative treatment strategies will enable hydrogel and nanotechnology-based approaches to revolutionize OA management, significantly improving patient outcomes and offering a new standard in joint health and repair.

## Data Availability

Data sharing is not applicable to this article as no new data were created or analyzed in this study.
